The article "Analysis of the Application Value of Ultrasound Three-Dimensional Speckle Tracking Technology Combined with Thyroid Autoantibodies and Hormones in the Diagnosis and Treatment of Graves' Disease" was retracted in 2023. Reasons: unreliable results or conclusions; concerns about the data; concerns about the peer review; concerns about the citations.

# Analysis of the Application Value of Ultrasound Three-Dimensional Speckle Tracking Technology Combined with Thyroid Autoantibodies and Hormones in the Diagnosis and Treatment of Graves' Disease

**DOI:** 10.1155/2022/7774283

**Published:** 2022-07-06

**Authors:** Yi Xu, Songxia Peng, Li Qin, Dianjing Sun, Jianlin Geng, Qingqing Liu

**Affiliations:** ^1^Endocrine Department, Hengshui People's Hospital, Hengshui, Hebei, China; ^2^The Second Department of Ultrasound, Hengshui People's Hospital, Hengshui, Hebei, China

## Abstract

**Objective:**

The aim of the study is to evaluate the application value of three-dimensional speckle tracking imaging (3D-STI) and combined detection of thyroid autoantibodies and hormones in the diagnosis and treatment of Graves' disease.

**Methods:**

A total of 60 patients with Graves' disease enrolled in our hospital from February 2020 to February 2021 were included in the experimental group, and 60 healthy patients after a physical examination during the same period were selected as the control group. No intervention was performed on the control group, and the experimental group received conventional Graves' disease treatment. The levels of thyroid autoantibodies and hormones in the two groups before and after the treatment were measured, and the 3D-STI was performed to compare the 3D-STI strain parameters of the research objects.

**Results:**

A significantly higher level of thyroid autoantibodies in the experimental group than that in the control group before and after the treatment was found (*P* < 0.001), with a remarkable decline observed after the treatment (*P* < 0.001). The positive rate of thyroid autoantibodies in the experimental group before the treatment was significantly higher than that in the control group (*P* < 0.05). After the treatment, the positive rate of TRAb and TPOAb was higher than that of the control group (*P* < 0.05), and the positive rate of TPOAb was higher than before the treatment. The two groups showed no significant difference in the positive rate of TGAb (*P* > 0.05). Significant differences were observed in the thyroid hormone levels between the two groups and also between before and after the treatment (*P* < 0.001). The experimental group garnered significantly higher 3D-STI strain parameters than the control group before the treatment (*P* < 0.05); after the treatment, the hyperthyroidism of the patients was relieved with a decreased 3D-STI value, but it was still notably higher than the control group (*P* < 0.05). Remarkably higher positive rates of combined detection before and after the treatment in the experimental group than those in the control group were obtained (*P* < 0.05).

The article "Analysis of the Application Value of Ultrasound Three-Dimensional Speckle Tracking Technology Combined with Thyroid Autoantibodies and Hormones in the Diagnosis and Treatment of Graves' Disease" was retracted in 2023. Reasons: unreliable results or conclusions; concerns about the data; concerns about the peer review; concerns about the citations.

**Conclusion:**

The combined detection of 3D-STI and thyroid autoantibodies and hormones ensures a better detection rate of Graves' disease and monitors the treatment effect of patients in real time, which provides a basis for clinical diagnosis and treatment and merits clinical promotion and application.

## 1. Introduction

Graves' disease is the most common organ-specific autoimmune disorder of primary hyperthyroidism, causing abnormalities in thyroid hormone secretion and involving multiple organ systems throughout the body, with a probability of more than 80% damage to the cardiovascular system [1], and most patients also often have concomitant proptosis, eyelid oedema, and reduced vision. Many studies suggest that there is a strong genetic link to the disease. Sequential cases of the disease are often seen in families, mostly in women [2]. The development of hyperthyroidism is significantly associated with human leukocyte antigens (HLA class II antigens), the detection rate of which varies according to ethnicity [3]. This may be due to a dramatic increase in adrenocorticotropic hormone production during high stress, which alters the function of suppressor T lymphocytes (Ts), or helper T lymphocytes (Th), thereby enhancing the immune response [4]. Patients are prone to cardiomyopathy and even heart failure in the advanced stages of the disease [5, 6], which can be life-threatening. For patients with Graves' disease, iodine is the main element in the production of thyroid hormones, and excessive intake by patients can make the condition worse or prolonged. Therefore, iodine is absolutely forbidden in patients with Graves' disease, as is the consumption of salt-containing iodine and related seafood. Patients with Graves' disease are very susceptible to vitamin deficiencies, so first of all, it is advisable for patients to eat fresh vegetables and fruit to get enough vitamins, or for those who have difficulty absorbing them, to take vitamin preparations directly.

Advanced research on the diagnosis and treatment of Graves' disease can effectively improve the prognosis of patients. To date, it has been shown that thyroid autoantibodies and hormones show great potential in the detection of Graves' disease [7–10]; however, such tests do not reflect the patient's functional impairment and compromise the objectivity of the functional evaluation of the treatment centre. Testing in combination with other diagnostic measures is therefore of great importance. Chest radiographs and echocardiography are commonly used in clinical practice to examine cardiac function [11]. Chest radiographs fail to evaluate abnormal cardiac function in patients in the early stages of the disease and have low sensitivity, while echocardiography is influenced by subjective factors and the reproducibility of cardiac function indicators obtained is suboptimal [12]. In recent years, two-dimensional scatter tracking imaging has been used in a variety of cardiac-related diseases, without angular dependence, to track frame by frame the acoustic scatter of left ventricular myocardial motion during the cardiac cycle. Three-dimensional speckle tracking imaging (3D-STI) is a convenient, rapid, and reproducible method for evaluating the longitudinal, radial, and circumferential strain of the LV myocardium and is a promising tool for evaluating ventricular wall motion, as it is more time-efficient and efficient than two-dimensional speckle tracking imaging in terms of image acquisition and offline analysis [13]. 3D-STI further modifies the disadvantages of planar imaging by providing a clear picture of the three-dimensional motion of the heart. The 3D-STI further changes the drawbacks of planar imaging and clearly presents the three-dimensional motion of the heart, providing a basis for the diagnosis and treatment of coronary stenosis and coronary heart disease [14–16].

The article "Analysis of the Application Value of Ultrasound Three-Dimensional Speckle Tracking Technology Combined with Thyroid Autoantibodies and Hormones in the Diagnosis and Treatment of Graves' Disease" was retracted in 2023. Reasons: unreliable results or conclusions; concerns about the data; concerns about the peer review; concerns about the citations.

Currently, few scholars have been able to draw on any systematic research into the application of 3D-STI in the diagnosis and treatment of Graves' disease. Accordingly, this study explored the application value of 3D-STI combined with thyroid autoantibodies and hormones. The report is as follows.

## 2. Materials and Methods

### 2.1. General Information

A total of 60 patients with Graves' disease enrolled in our hospital from February 2020 to February 2021 were included in the experimental group, and 60 healthy patients after a physical examination during the same period were selected as the control group. This study was approved by the ethics committee of the hospital.

### 2.2. Inclusion Criteria

The patients are included if (1) the patients or their family members signed the informed consent form after being fully informed of the purpose and process of the study; (2) the patients were diagnosed with Graves' disease after laboratory examination and clinical diagnosis [17]; and (3) the patients had symptoms and signs of hyperthyroidism and diffuse thyroid enlargement [18].

### 2.3. Exclusion Criteria

The patients (1) with mental problems or inability to communicate; (2) with other organic diseases, including other thyroid diseases; (3) with a history of endocrine diseases; and (4) who received treatment for Graves' disease within one month before admission [19, 20]are excluded.

### 2.4. Method

#### 2.4.1. 3D-STI

A three-dimensional probe of a color Doppler ultrasound diagnostic equipment (GE medical color ultrasound diagnostic equipment Voluson P6, National Machinery Injection 20152062178) was used to obtain a four-chamber view of the apex of the heart, configured with the three-dimensional probe X5-1, with the frequency of 2.0–3.8 MHz and external three-dimensional analysis software (Imaging Systems, Munich, Germany). With the loop of 1, the patients were instructed to hold their breath to obtain a two-dimensional image, and then the full volume mode was employed to collect the dynamic raw data of three consecutive stable cardiac cycles when the subject holds their breath at the end of the expiration. All the images were copied into the workstation for 3D-STI analysis by using the 3D analysis software.

The article "Analysis of the Application Value of Ultrasound Three-Dimensional Speckle Tracking Technology Combined with Thyroid Autoantibodies and Hormones in the Diagnosis and Treatment of Graves' Disease" was retracted in 2023. Reasons: unreliable results or conclusions; concerns about the data; concerns about the peer review; concerns about the citations.

Real-time volumetric image import: Based on clear endocardial and epicardial images of the left ventricular wall, positioned at the midpoint of the mitral valve and the apical part of the left ventricle, with the tip of the *P* wave as the end-diastolic phase and the end of the *T* wave as the systolic phase, the program observes the end-diastolic and end-systolic left ventricular membrane curves displayed and comprehensively tracks the movement of myocardial patches. Left ventricular global longitudinal strain (GLS), left ventricular global circumferential strain (GCS), left ventricular twist (LV-tw), left ventricular torsion (LV-tor), left ventricular peak basal rotation (Prot-B), left ventricular peak apical rotation (Prot-A), and left ventricular ejection fraction (LVEF) were calculated.

#### 2.4.2. Thyroid Autoantibody and Hormone Detection

The fasting venous blood before and after the treatment was drawn from the patients, and the serum was separated after 2 hours of standing in the blood collection tube. Chemiluminescence immunoassay (Cubase 411 electrochemiluminescence instrument, original supporting reagents, NMPA Approval No. 3402843) was used to determine the levels of thyroid hormone receptor antibody (TRAb), thyroid peroxidase antibody (TPOAb), and thyroglobulin antibody (TGAb). Serum-free triiodothyronine (FT3), serum-free thyroxine (FT4), and thyroid-stimulating hormone (TSH) levels were measured using a particulate chemiluminescence method (Myriad CL-2000i, original companion reagent, NMPA Standard 2013 No. 3401028).

#### 2.4.3. Treatment

All patients were treated with methimazole (Beijing Taiyang Pharmaceutical Co. Ltd., Zhunzi H11020885), orally at 30–40 mg/d, and the dosage was gradually decreased according to the clinical symptoms and thyroid function. The treatment lasted for 12 weeks.

### 2.5. Observational Criteria

1. Thyroid autoantibody level [21]: TRAb, TPOAb, and TGAb. The normal range for TRAb is 0 to 1.75 IU/L; for TPOAb, 0 to 60 U/mL; and for TgAb, 0 to 100 IU/mL. Positivity rate = number of people who tested positive at test level/total number of people.
2. Thyroid hormone levels [22]: FT3, FT4, and TSH. The normal range for TSH is 0.55 to 4.78 µIU/mL; the normal range for free T4 is 0.89 to 1.76 ng/dL; and the normal range for T3 is 60 to 181 ng/dL.
3. 3D-STI strain parameters: GLS, GCS, LV-tw, LV-tor, Prot-B, Prot-A, LVEF, left ventricular end-diastolic volume (LVEDV), and left ventricular end-systolic volume (LVESV).
4. The positive rate of combined detection of 3D-STI and thyroid autoantibodies and hormones was calculated. Positivity rate = number of people who tested positive at test level/total number of people.

The article "Analysis of the Application Value of Ultrasound Three-Dimensional Speckle Tracking Technology Combined with Thyroid Autoantibodies and Hormones in the Diagnosis and Treatment of Graves' Disease" was retracted in 2023. Reasons: unreliable results or conclusions; concerns about the data; concerns about the peer review; concerns about the citations.

### 2.6. Withdrawal Criteria

The withdrawal criteria are as follows: (1) the patients with adverse events or serious adverse events, (2) the patients with condition deteriorated during the experiment, (3) the patients with serious comorbidities or complications, and (4) the patients who were unwilling to continue the clinical trial and asked for withdrawal.

Regardless of the above reasons, for the cases who withdrew from the trial, their records were retained, with the last test results as the final results for data analysis.

### 2.7. Statistical Processing

The data obtained in this study were processed by software SPSS20.0, and the graphics plotting was processed using GraphPad Prism 7 (GraphPad Software, San Diego, USA) software. The research data included count data and measurement data. Count data were processed by the X2 test, and the measurement data were analyzed by *t*-test. *P* < 0.05 indicates statistical significance.

## 3. Results

### 3.1. General Information

The two groups showed no significant difference in general information (*P* > 0.05; see Table 1).

### 3.2. Comparison of Thyroid Autoantibody Levels

The pre-treatment (37.21 ± 5.22) and post-treatment (25.15 ± 2.41) levels of TRAb in the experimental group were significantly higher than those in the control group (11.98 ± 1.22, 11.98 ± 1.22), and the pre-treatment levels of TRAb in the experimental group were significantly higher than those after the treatment (*P* < 0.001). The pre-treatment (69.65 ± 5.14) and post-treatment (45.26 ± 3.54) TPOAb levels in the experimental group were significantly higher than those in the control group (26.54 ± 3.21, 26.54 ± 3.21), and the pre-treatment TRAb levels in the experimental group were significantly higher than those after the treatment (*P* < 0.001). The pre-treatment (28.98 ± 20.11) and post-treatment (13.68 ± 10.14) TGAb levels in the experimental group were significantly higher than those in the control group (5.10 ± 4.98, 5.10 ± 4.98), and the pre-treatment TGAb levels in the experimental group were significantly higher than those after the treatment (*P* < 0.001; see Figure 1).

The article "Analysis of the Application Value of Ultrasound Three-Dimensional Speckle Tracking Technology Combined with Thyroid Autoantibodies and Hormones in the Diagnosis and Treatment of Graves' Disease" was retracted in 2023. Reasons: unreliable results or conclusions; concerns about the data; concerns about the peer review; concerns about the citations.

The pre-treatment thyroid autoantibody positivity rate was significantly higher in the experimental group (60%) than in the control group (8.3%; *P* < 0.05). The post-treatment rate of TRAb and TPOAb positivity remained higher than that of the control group (41.7% vs. 8.3%; *P* < 0.05), and the TPOAb positivity rate was higher than that before treatment. The TGAb positivity rate decreased in the experimental group after treatment (60% vs. 41.7%), while the difference in TGAb positivity rate between the two groups was not statistically significant (*P* > 0.05), as shown in Figures 2–4.

### 3.3. Comparison of Thyroid Hormone Levels

FT3 levels in the experimental group were higher before treatment (14.21 ± 2.10) than after treatment (5.98 ± 1.04), and both were higher than in the control group (2.98 ± 1.00). FT4 levels in the experimental group were higher before treatment (45.68 ± 3.65) than after treatment (24.55 ± 3.10), and both were higher than in the control group (11.54 ± 2.10). TSH levels in the experimental group were higher before treatment (0.012 ± 0.003) than after treatment (0.310 ± 0.105), and both were higher than in the control group (2.340 ± 1.211). Significant differences were observed in the thyroid hormone levels between the two groups and also between before and after the treatment (*P* < 0.001; see Table 2).

### 3.4. Comparison of 3D-STI Strain Parameters

The experimental group garnered significantly higher 3D-STI strain parameters than the control group before the treatment (*P* < 0.05); after the treatment, the hyperthyroidism of the patients was relieved with a decreased value, but it was still significantly higher than the control group (*P* < 0.05; see Table 3).

### 3.5. Comparison of Positive Rates of Combined Detection

There were 58 positive cases (96.7%) in the experimental group before treatment, 54 positive cases (90.0%) after treatment, and 1 positive case (1.7%) in the control group. Remarkably higher positive rates of combined detection before and after the treatment in the experimental group than those in the control group were observed (*P* < 0.05; see Figure 5).

## 4. Discussion

Studies in recent decades have confirmed the close relation of the occurrence of hyperthyroidism to thyroid autoantibody stimulation of the thyroid [23–26]. TPOAb and TGAb are both destructive antibodies with their target antigens of thyroid peroxidase and thyroglobulin, respectively. They work together to form an immune response to thyroid antigens and lead to the release of thyroid hormones to induce hyperthyroidism secondary to antibody-dependent cell-mediated cytotoxicity that destroys thyroid follicles. TRAb, the most important type of stimulating antibody related to hyperthyroidism, activates the cAMP pathway by acting on the TSH receptor of thyroid cells, accelerates the proliferation of thyroid cells, and increases the frequency of synthetic thyroid hormone secretion, eventually giving rise to Graves' disease [27, 28]. Many studies have shown that Graves' disease can easily be confused with other conditions and lead to misdiagnosis if only thyroid autoantibody and hormone levels are tested [29]. Simple goitre, in addition to goitre, is mostly shown to be suppressible by T3 suppression tests, although 131I uptake is sometimes increased [30]. Hashimoto's disease is also an autoimmune disease similar to Graves' disease [31]. There are also many patients with mild disease or elderly and paediatric cases with few and atypical clinical presentations, which are also difficult to detect accurately.

The article "Analysis of the Application Value of Ultrasound Three-Dimensional Speckle Tracking Technology Combined with Thyroid Autoantibodies and Hormones in the Diagnosis and Treatment of Graves' Disease" was retracted in 2023. Reasons: unreliable results or conclusions; concerns about the data; concerns about the peer review; concerns about the citations.

In this study, the level of thyroid autoantibodies in the experimental group was significantly higher than that in the control group before and after the treatment (*P* < 0.001), despite a remarkable decline observed after the treatment (*P* < 0.001), indicating the close relation between the occurrence and development of Graves' disease to thyroid autoantibodies and hormones that show great potential in the diagnosis of the disease. In the study by Liew et al., the positive rate of TRAb in diagnosing Graves' disease was 55% [32]. This study showed that the positive rate of the antibody in diagnosing Graves' disease was 60%. After the treatment, the positive rate of TRAb dropped to 41.7%, which demonstrated that TRAb can reflect the degree of the patient's disease yet fails to exert a decisive effect on the diagnosis and treatment of the disease. Apart from TRAb, changes in the patient's antibody indicators with the remission of the disease have also been witnessed. After the treatment, the positive rate of TRAb and TPOAb was still higher than that of the control group (*P* < 0.05), and the positive rate of TPOAb was higher than before the treatment. The two groups showed no significant difference in the positive rate of TGAb (*P* > 0.05). Despite the different trends in the three antibodies, it is noteworthy that FT3 and FT4 showed a steady decline, indicating improved cardiac function; however, thyroid autoantibodies and hormone levels are not sufficient as an objective basis for reflecting cardiac indicators and other tests are needed [33, 34].

In light of heart involvement, thyroid hormone strengthens the contractility of the myocardium by directly acting in the heart or affecting the sympathetic nerve. The accelerated heart rate and the shortened cardiac cycle may develop cardiomyopathy under the effect of autoimmune injuries, with main manifestations of enhanced overall systolic function of the left ventricle in the early stage and decreased myocardial contraction and active relaxation force in the advanced stage. Imaging is used clinically to monitor changes in patients with Graves' disease as described above and to provide a basis for the diagnosis of the disease. 3D-STI is a new inspection method that has emerged in recent years. It allows frame-by-frame tracking of the acoustic spot of left ventricular myocardial motion during the cardiac cycle, regardless of angle, and accurately reflects the complex three-dimensional motion of the heart. Due to the specific structure of the left ventricular wall myocardium, three patterns of cardiac motion are identified during the mechanical activity of the myocardium, including longitudinal, circular, and radial [35]. The torsional movement of the heart is closely related to the contraction function. The myocardium under the endocardium of the left ventricle receives the greatest force, and the systolic displacement in the long axis direction of the myocardium decreases rapidly, which contributes to the increasing trend of 3D-STI strain parameters. After the treatment, the hyperthyroidism of the patients was relieved with a decreased 3D-STI value, but it was still significantly higher than the control group (*P* < 0.05), indicating the potential of 3D-STI in the evaluation of cardiac function. The positive rate of this examination method combined with thyroid autoantibodies and hormones was significantly higher than that of the control group (*P* < 0.05), verifying the improvement of the accuracy of clinical diagnosis and treatment.

The article "Analysis of the Application Value of Ultrasound Three-Dimensional Speckle Tracking Technology Combined with Thyroid Autoantibodies and Hormones in the Diagnosis and Treatment of Graves' Disease" was retracted in 2023. Reasons: unreliable results or conclusions; concerns about the data; concerns about the peer review; concerns about the citations.

Traditional treatment options carry the risk of disease recurrence, lifelong thyroid hormone replacement therapy, and complications, while other new treatment options have limitations. A study has shown that herbal medicine is an effective alternative for the treatment of hyperthyroidism due to Graves' disease, especially in patients with an allergy to thionamide [36]. When used as an adjunctive medicine, the active ingredients of herbal medicine are not only effective in relieving goitre, Graves' ophthalmopathy symptoms, and hypermetabolic symptoms but also in reducing the side effects and allergic symptoms of antithyroid drugs and in increasing the dose of ATD in allergic patients [37]. There is now a need to expand the understanding of how Chinese medicine can help in the treatment of Graves' disease. Some herbs used in combination with antithyroid drugs can induce apoptosis (removal of excess tissue from the thyroid gland), and herbal medicine has been shown to be a valuable adjunct to the normal treatment of Graves' disease, particularly in patients who have antithyroid drug side effects and do not wish to start radioactive iodine therapy [38]. Therefore, in combination with the results of this study and the above, the use of Western diagnostic modalities combined with TCM treatment modalities may become a new clinical direction for Graves' disease in the future.

In conclusion, the combined detection of 3D-STI and thyroid autoantibodies and hormones ensures a better detection rate of Graves' disease and monitors the treatment effect of patients in real-time, which provides a basis for clinical diagnosis and treatment and merits clinical promotion and application. However, our study sample and selection should be expanded in subsequent experiments to a more broad-spectrum study, and given the inadequate sample size for statistical measurements, regional errors may occur. And the response is a long-term process, for prognosis also issues should be designed into future experiments.

## Figures and Tables

**Figure 1:** Comparison of thyroid autoantibody levels of study subjects ($\bar{x}$ ± *s*, %). The abscissa from left to right is the control group, the experimental group before treatment, and the experimental group after treatment, respectively. ^#^*P* < 0.001. (a) TRAb level. The TRAb level of the experimental group before and after treatment was significantly higher than that of the control group (37.21 ± 5.22 vs. 11.98 ± 1.22, 25.15 ± 2.41 vs. 11.98 ± 1.22, *P* < 0.001); the level of TRAb in the experimental group before treatment was significantly higher than after treatment (37.21 ± 5.22 vs. 25.15 ± 2.41, *P* < 0.001). (b) TPOAb level (%). The TPOAb level of the experimental group before and after treatment was significantly higher than that of the control group (69.65 ± 5.14 vs. 26.54 ± 3.21, 45.26 ± 3.54 vs. 26.54 ± 3.21, *P* < 0.001); the level of TPOAb was significantly higher than after treatment (69.65 ± 5.14 vs. 45.26 ± 3.54, *P* < 0.001). (c) TGAb level (%). The TGAb level of the experimental group before and after treatment was significantly higher than that of the control group (28.98 ± 20.11 vs. 5.10 ± 4.98, 13.68 ± 10.14 vs. 5.10 ± 4.98, *P* < 0.001); the level of TGAb was significantly higher than after treatment (28.98 ± 20.11 vs. 13.68 ± 10.14, *P* < 0.001).

**Figure 2:** Comparison of TRAb positive rate (*n* (%)). The black area is positive, and the gray area is negative; the left, middle, and right are the experimental group before treatment, the experimental group after treatment, and the control group, respectively. ^#^*P* < 0.05.

The article "Analysis of the Application Value of Ultrasound Three-Dimensional Speckle Tracking Technology Combined with Thyroid Autoantibodies and Hormones in the Diagnosis and Treatment of Graves' Disease" was retracted in 2023. Reasons: unreliable results or conclusions; concerns about the data; concerns about the peer review; concerns about the citations.

**Figure 3:** Comparison of TPOAb positive rate (*n* (%)). The black area is positive, and the gray area is negative; the left, middle, and right are the experimental group before treatment, the experimental group after treatment, and the control group, respectively. ^#^*P* < 0.05.

**Figure 4:** Comparison of TGAb positive rate (*n* (%)). The black area is positive, and the gray area is negative; the left, middle, and right pie charts are the experimental group before treatment, the experimental group after treatment, and the control group, respectively. ^#^*P* < 0.05. The positive rate of TGAb in the experimental group before treatment was significantly higher than that in the experimental group after treatment and the control group (36 vs. 12, 36 vs. 5, *P* < 0.05).

**Figure 5:** Comparison of positive rates of combined detection (*n* (%)). The abscissa is, from left to right, the experimental group before treatment, the experimental group after treatment, and the control group. The ordinate is positive patients (cases). ^#^*P* < 0.05. The number of positive cases in the experimental group before treatment was 58 (96.7%); the number of positive cases after treatment was 54 (90.0%); and the number of positive cases in the control group was 1 (1.7%).

**Table 1:** Comparison of general information of patients.

Groups	Experimental group (*n* = 60)	Control group (*n* = 60)	*X* ^2^/*t*	*P*
Gender			0.037	0.847
Male	20	21		
Female	40	39		
Age (year)				
Range	35–60	36–60		
Average age	46.21 ± 2.65	46.32 ± 2.41	0.043	0.967
Average weight (kg)	54.68 ± 1.65	54.58 ± 1.58	0.339	0.735
BMI (kg/m^2^)	22.54 ± 1.22	22.36 ± 1.23	0.805	0.423
Place of residence			0.034	0.855
Urban	32	33		
Rural	28	27		
Monthly income (year)			0.133	0.715
≥4,000	31	29		
<4,000	29	31		
Living habits				
Smoking	29	28	0.033	0.855
Drinking	32	33	0.034	0.855
Education level			0.033	0.855
High school and below	30	29		
Junior college and above	30	31		

**Table 2:** Comparison of thyroid hormone levels ($\bar{x}$ ± *s*).

Groups	Experimental group		Control group
	Before treatment	After treatment	
FT3	14.21 ± 2.10^*∗*^^#^	5.98 ± 1.04^#^	2.98 ± 1.00
FT4	45.68 ± 3.65^*∗*^^#^	24.55 ± 3.10^#^	11.54 ± 2.10
TSH	0.012 ± 0.003^*∗*^^#^	0.310 ± 0.105^#^	2.340 ± 1.211

^*∗*^Compared with after treatment, *P* < 0.001; ^#^compared with the control group, *P* < 0.001.

**Table 3:** Comparison of 3D-STI strain parameters ($\bar{x}$ ± *s*).

Parameters	Experimental group		Control groups
	Before treatment	After treatment	
GLS (%)	−22.65 ± 2.10^*∗*^^#^	−19.98 ± 2.11^#^	−17.68 ± 1.20
GCS (%)	−30.32 ± 2.98^*∗*^^#^	−27.54 ± 2.14^#^	−24.98 ± 2.65
LV-tw (°)	16.54 ± 5.21^*∗*^^#^	14.26 ± 4.65^#^	9.89 ± 5.41
LV-tor (°/cm)	2.10 ± 0.67^*∗*^^#^	1.79 ± 0.68^#^	1.29 ± 0.45
Prot-b (°)	−9.12 ± 2.35^*∗*^^#^	−8.12 ± 2.12^#^	−6.54 ± 2.65
Prot-a (°)	7.10 ± 3.41^*∗*^^#^	5.54 ± 3.11^#^	4.24 ± 3.68
LVEF (%)	60.21 ± 2.15^*∗*^^#^	56.68 ± 2.65^#^	55.68 ± 1.23
LVEDV (mL)	115.68 ± 12.65^*∗*^^#^	108.65 ± 12.21^#^	97.65 ± 15.22
LVESV (mL)	50.65 ± 6.98^*∗*^^#^	46.98 ± 5.44^#^	42.98 ± 5.41

^*∗*^Compared with after treatment, *P* < 0.05; ^#^compared with the control group, *P* < 0.05.

The article "Analysis of the Application Value of Ultrasound Three-Dimensional Speckle Tracking Technology Combined with Thyroid Autoantibodies and Hormones in the Diagnosis and Treatment of Graves' Disease" was retracted in 2023. Reasons: unreliable results or conclusions; concerns about the data; concerns about the peer review; concerns about the citations.

## Data Availability

All data generated or analyzed during this study are included in this published article.
